The article "Laparoscopic Port Site Hernia: A Rare Etiology of Intestinal Obstruction" was retracted in 2024. Reasons: false authorship; unreliable results or conclusions; no approval from an author; concerns about the authorship.

# Laparoscopic Port Site Hernia: A Rare Etiology of Intestinal Obstruction

**DOI:** 10.7759/cureus.19681

**Published:** 2021-11-17

**Authors:** Alanood M Albaqami, Hawra’a A Al-Salam, Mona A Alhagbani, Rahmah A Fallatah, Abdullah M Aljarboa, Majed A Alghassab, Saeed S Alghamdi, Kawthar A Kadhem, Yahya T Alsaileek, Hussam A Albarakati, Ziyad I Gadah, Abdulqader S Babhair, Mohammad Y Alshammari, Masooma A Abuidrees, Faisal M Al-Hawaj

**Affiliations:** 1 College of Medicine, Dar Al Uloom University, Riyadh, SAU; 2 College of Medicine, University of Hail, Hail, SAU; 3 College of Medicine, Al-Baha University, Al-Baha, SAU; 4 Family Medicine, Dammam Medical Complex, Dammam, SAU; 5 College of Medicine, Imam Abdulrahman Bin Faisal University, Dammam, SAU; 6 College of Medicine, Umm Al-Qura University, Mecca, SAU; 7 College of Medicine, King Abdulaziz University, Jeddah, SAU; 8 College of Medicine, Arabian Gulf University, Manama, BHR; 9 Family Medicine, King Khalid University Hospital, Riyadh, SAU

**Keywords:** case report, port-site hernia, laparoscopy, intestinal obstruction, hernia, acute abdominal pain

## Abstract

Small intestinal obstruction is a common indication for hospitalization and emergency surgeries. The most frequent etiologies are adhesions, hernia, and benign or malignant neoplasms. Abdominal imaging plays an important role in making the diagnosis and evaluating the complications of the obstruction. We report a case of a young woman who presented with sudden abdominal pain and vomiting. She had a relevant past medical history of sickle cell disease and multiple episodes of biliary colic for which she underwent laparoscopic cholecystectomy two months before her current presentation. Laboratory findings indicated mild inflammation in the form of elevated C-reactive protein and erythrocyte sedimentation rate with the leukocytes count in the upper normal limits. Abdominal computed tomography demonstrated a knuckle of small bowel incarcerated in the port location of the previous laparoscopy. The bowel was reduced and the defect was repaired. The patient had complete resolution of her symptoms following the surgery. The case highlighted the importance of considering port-site hernia as an etiology of bowel obstruction in the relevant clinical settings since laparoscopic operations are being increasingly performed.

## Introduction

Acute intestinal obstruction is a common surgical emergency. It accounts for 15% of admissions and 20% of emergency abdominal surgeries [1]. Intestinal obstruction can be mechanical or functional. The mechanical obstruction can be caused by intraluminal or extraluminal compression. In developed countries, adhesion is the most common cause of small intestinal obstruction [1]. Indeed, the small intestinal obstruction is due to adhesions, hernia, or neoplasm in more than 90% of cases [2]. While the diagnosis of small intestinal obstruction can be suspected by its clinical features, abdominal imaging is essential to make the diagnosis and obtain more details about the obstruction, including its location, severity, complication, and the possible underlying cause. Here, we present a case of a young woman who presented with a clinical picture suggestive of intestinal obstruction and was found to have a laparoscopic port-site hernia, a very rare etiology of intestinal obstruction.

The article "Laparoscopic Port Site Hernia: A Rare Etiology of Intestinal Obstruction" was retracted in 2024. Reasons: false authorship; unreliable results or conclusions; no approval from an author; concerns about the authorship.

## Case presentation

Our patient is a 34-year-old woman who presented to the emergency department because of abdominal pain for two days duration. The pain was generalized and colicky in nature with no radiation. It was not related to meal intake. She used over-the-counter analgesic and antispasmodics agents and had no improvement in her pain. She rated the pain as 8 on the 10-point severity scale and reported that it has been increasing in severity. The pain was associated with nausea and recurrent episodes of vomiting. She reported a history of constipation and decreased appetite. She did not experience similar pain episodes previously. The patient is known to have sickle cell disease and had undergone laparoscopic cholecystectomy two months before due to recurrent episodes of biliary colic. The operation was not eventful for any complications. Her medication includes hydroxyurea for sickle cell disease. She worked as a pediatric nurse. She was a non-smoker and had never consumed alcohol. The family history is remarkable for inflammatory bowel disease.

Upon examination, the patient appeared in pain with no signs of respiratory distress. Her vital signs showed tachycardia (107 bpm), tachypnea (21 bpm), normal temperature (37.3℃), and maintained blood pressure (115/80 mmHg). The oxygen saturation was 98% on room air. Abdominal examination revealed a soft abdomen with generalized tenderness. No guarding or rigidity was noted. Bowel sounds were increased in intensity and frequency. It was noted that the skin overlying the incision was warm and tender. Examination of the hernial orifices was normal. Cardiorespiratory examination revealed normal findings. Initial laboratory investigation revealed a hemoglobin level of 14.2 g/dL, leukocyte count of 11,000/μL, and platelet count of 380,000/μL. C-reactive protein and erythrocyte sedimentation rates were mildly elevated. Further, the renal profile showed mild elevation in blood urea nitrogen level. The remainder of the laboratory findings, including electrolytes and hepatic profile, were within the reference ranges (Table 1).

The article "Laparoscopic Port Site Hernia: A Rare Etiology of Intestinal Obstruction" was retracted in 2024. Reasons: false authorship; unreliable results or conclusions; no approval from an author; concerns about the authorship.

**Table 1:** Summary of the results of laboratory findings.

Laboratory investigation	Unit	Result	Reference range
Hemoglobin	g/dL	14.2	13.0–18.0
Leukocytes	1000/mL	11.0	4.0–11.0
Platelet	1000/mL	380	140–450
C-reactive protein	mg/dL	13.3	0.3–10.0
Erythrocyte sedimentation rate	mm/hr.	25	0–20
Albumin	g/dL	3.9	3.4–5.0
Total bilirubin	mg/dL	0.8	0.2–1.2
Alanine transferase	U/L	52	14–63
Aspartate transferase	U/L	21	15–37
Gamma-glutamyltransferase	U/L	65	15–85
Alkaline phosphatase	U/L	80	46–116
Creatinine	mg/dL	0.9	0.7–1.3
Blood urea nitrogen	mg/dL	15	7–18
Serum sodium	mEq/L	138	136–145
Serum potassium	mEq/L	3.6	3.5–5.1
Serum chloride	mEq/L	104	98–107

In light of the aforementioned details, an abdominal computed tomography scan with intravenous contrast was performed. The scan demonstrated multiple distended loops of the small bowel with a transition point in the midline of the abdomen. No signs of bowel ischemia were noted. A small amount of intraperitoneal fluid was observed. No pneumoperitoneum was seen. The abdominal wall was edematous and a knuckle of the small bowel was seen herniating through the trocar site of the previous laparoscopic surgery. Such findings were representing a small intestinal obstruction secondary to hernia through the trocar site (Figure 1).

**Figure 1:** Axial (A) and sagittal (B) CT images demonstrating a knuckle of the small bowel herniating through an anterior abdominal wall (arrow) with surrounding subcutaneous edema.

Subsequently, the patient was resuscitated with intravenous fluid. Intravenous lornoxicam 8 mg was given for pain control. The patient was planned to undergo emergency laparoscopy for reduction of the incarcerated hernia. The operation was done under general anesthesia. The patient was placed in a supine position. After inserting the trocars and establishing the pneumoperitoneum, a diagnostic evaluation was conducted. The laparoscopic findings confirmed the radiological findings, in which a small intestinal loop was seen herniating through the trocar site of previous surgery. Reduction of the intestinal loop was made and the defect was repaired. No complications occurred during the operation. The operative time was 60 minutes. No significant blood loss was noted. The recovery of the patient was uneventful. Following the surgery, the patient tolerated oral feeding. She was discharged four days following the surgery. Six weeks later, the patient was seen in the clinic with no active complaints.

## Discussion

We presented the case of a port-site hernia with acute small intestinal obstruction. Such complication is one of the major complications of laparoscopic surgeries, but it is very rare and requires a high index of suspicion [3]. In a review of reported cases in the literature, Boughey et al. [4] reported that the incidence of port-site hernia is less than three per 1,000 cases. As in our case, the port-site hernia may be associated with complications, such as incarceration and bowel obstruction.

The article "Laparoscopic Port Site Hernia: A Rare Etiology of Intestinal Obstruction" was retracted in 2024. Reasons: false authorship; unreliable results or conclusions; no approval from an author; concerns about the authorship.

Some patient and operation factors have been reported to increase the likelihood of developing port-site hernia [5]. Obesity and diabetes mellitus were among the most important patient’s related risk factors [3]. Regarding the surgery factors, it was found that extensive manipulation of the trocar during the operation increases the risk of herniation by increasing the trocar site size [4]. Further, the port-site hernia is more common when a non-bladed trocar is used. In the present case, a non-bladed trocar was used. Some authors suggested that leaving the fascial defect open raises the possibility of future port-site hernia [6]. In the present case, the fascial defect was not closed, which may predispose the patient to port-site herniation.

The clinical manifestation of port-site herniation varies depending on the degree of bowel obstruction. It may present with mild nausea and abdominal discomfort [3]. In contrast, it may present with acute abdominal as in the present case. Considering its non-specific presentation, the diagnosis of port-site hernia may be delayed [6]. Additionally, the hernia can have an early or late presentation. A computed tomography scan can establish the diagnosis accurately.

## Conclusions

The port-site hernia is a rare yet serious complication of laparoscopic cholecystectomy. Physicians should keep this possible condition in their minds when they encounter a patient with clinical signs and symptoms of intestinal obstruction in patients with a recent or remote history of laparoscopic surgeries. A computed tomography scan is the investigation modality of choice to confirm the diagnosis.
